The article "Efficacy and Safety of Jinshuibao Capsule in Diabetic Nephropathy: A Systematic Review and Meta-Analysis of Randomized Controlled Trials" was retracted in 2023. Reasons: signs of a paper mill; compromised peer review; unreliable results or conclusions.

# Efficacy and Safety of Jinshuibao Capsule in Diabetic Nephropathy: A Systematic Review and Meta-Analysis of Randomized Controlled Trials

**DOI:** 10.1155/2022/9671768

**Published:** 2022-08-28

**Authors:** Xinyu Yu, Dongmei Yan, Qin Lan, Jianhe Fang, Zhaohui Ding, Yongmei Guan, Weifeng Zhu, Lei Yan, Heyun Nie

**Affiliations:** ^1^Center for Treatment of Diseases, Nanchang Hongdu Hospital of Traditional Chinese Medicine, Nanchang, Jiangxi Province, China; ^2^Academician Workstation, Jiangxi University of Jiangxi University of Traditional Chinese Medicine, Nanchang, Jiangxi Province, China; ^3^Evidence-Based Medicine Research Centre, Jiangxi University of Traditional Chinese Medicine, Nanchang, Jiangxi Province, China; ^4^The Affiliated Hospital of Jiangxi University of Jiangxi University of Traditional Chinese Medicine, Nanchang, Jiangxi Province, China; ^5^Key Laboratory of Modern Preparation of Traditional Chinese Medicine of Ministry of Education, Jiangxi University of Jiangxi University of Traditional Chinese Medicine, Nanchang, Jiangxi Province, China; ^6^Ophthalmology Department, Jiangxi Integrated Hospital of Traditional Chinese and Western Medicine, Nanchang, Jiangxi Province, China

## Abstract

**Objective:**

This systematic review was able to evaluate the clinical evidence of JSBC in the randomized controlled trial (RCT) of diabetic nephropathy.

**Methods:**

The Chinese and English literatures published in PubMed, Cochrane Library, VIP, Wanfang Data, CNKI, and CBM before July 30, 2019, were retrieved. This study includes only randomized controlled trials of treatments related to diabetic nephropathy. We assessed the methodological quality of the subjects involved according to the assessment criteria in 5.3.3 of the Cochrane Assessment Manual. RevMan 3.5.5 software was used to analyze the relevant data, meta-analysis, and inverted funnel analysis chart.

**Results:**

This study included 26 RCTs, including 4676 patients in total (2342 cases in the experimental group and 2334 cases in the control group). The results of 8 randomized controlled trials showed that urinary microprotein excretion rate (UAER) significantly decreased (*P* < 0.0001) before and after treatment of diabetic nephropathy.

**Conclusion:**

The available clinical evidence has suggested that JSBC combined with western drugs is differentially effective in the treatment of diabetic nephropathy. The combination of JSBC with western medicine is more effective. However, due to the small amount and low quality of the included literatures, the current evidence is not certain to be fully clinically applicable.

## 1. Introduction

Diabetic nephropathy is an important microvascular complication of diabetes and the main cause of death in diabetic patients. In developed countries such as the United States and the United Kingdom, renal failure caused by diabetic nephropathy has risen to the first place in end-stage renal disease [1]. In China, the incidence of diabetic nephropathy has been also up to 20-40% [1]. With the growing number of diabetic patients in China, the incidence of diabetic nephropathy is increasing year by year [2].

Clinically, diabetic nephropathy is characterized by glomerular mesangial cell proliferation, basement membrane thickening, or glomerulosclerosis. It lacks obvious clinical manifestations at the early stage. Therefore, early diagnosis is of great significance for the treatment of diabetes mellitus.

Jinshuibao belongs to Cs-4 preparation fermented Cordyceps sinensis powder, which is the extract of Cordyceps sinensis. It is further purified by modern Chinese medicine preparations. Its functions include invigorating the lungs and kidneys, draining essence and nourishing qi [3, 4]. Jinshuibao capsule (JSBC) is a common drug in clinical treatment of diabetic nephropathy. Urinary microprotein excretion rate (UAER) can reflect early nephropathy and renal injury. Therefore, it was regarded as the main outcome index in this paper.

In China, there are few studies on the efficacy of JSBC in the treatment of diabetic nephropathy. Therefore, this study is aimed at updating and critically evaluating the evidence from randomized controlled trials (RCTs) to examine the efficacy and safety of JSBC.

## 2. Materials and Methods

The study was conducted in accordance with the guidelines of PRISMA (Preferred Reporting Items for Systematic Reviews and Meta-Analyses).

### 2.1. Data Sources

The literature was retrieved through the following databases until August 2019, PubMed, Embase, the Cochrane Central Register of Controlled Trials, and four Chinese databases (WanFang Med Database, Chinese BioMedical Database, Chinese VIP Database, and China National Knowledge Infrastructure (CNKI)). Search strategies were listed in Table 1. In addition, the search terms were modified in different databases, based on the reference list of articles to all possible matching RCT-related titles.

### 2.2. Selection of Researches

This article was reviewed the efficacy of JSBC in the treatment of diabetic nephropathy in a RCT. Experiments published in the form of papers were also selected as eligible studies. All experiments met the following criteria and Picos principles (population, intervention, comparison, and results) without any language restrictions (Figure 1).

#### 2.2.1. P (Population)

The population matched the Megenson classification criteria. The clinical diagnosis of type 2 diabetic nephropathy was in the phase III.

#### 2.2.2. I (Intervention)

Twenty-six experiments were treated with JSBC alone, 18 experiments used JSBC combined with other drugs, and 8 experiments combined JSBC with basic drugs.

#### 2.2.3. C (Comparison)

The routine treatment of diabetic nephropathy patients in the control group should follow the consensus of experts on the prevention and treatment of diabetic nephropathy (2014 edition). The controlled cases were treated with biguanides, sulfonylureas, glinides, thiazolidinediones, d-mono-glycosidase inhibitors, dipeptidyl peptidase IV (DPP.4) inhibitors, glucagon-like peptide 1 (GLP.1) analogues, and insulin drugs. If therapeutic approach of control group was not related to the guidelines, the study would be excluded.

#### 2.2.4. O (Outcomes)

The core indicators of systematic evaluation included (1) urinary microprotein excretion rate, (2) urinary protein, (3) glycosylated hemoglobin, (4) urea nitrogen, (5) serum creatinine, and (6) fasting blood sugar.

### 2.3. Data Extraction, Quality, and Validation

All the literatures were screened by two researchers as per inclusion and exclusion criteria. The literature information was extracted, including the following aspects: (1) characteristics of study consisted of author (s), published year, study design, sample size, follow-up date, and efficacy criteria; (2) characteristics of patient consisted of patients' age, drug intervention and time of administration; (3) intervention measures included trial group intervention and control group intervention; (4) outcomes of study: two researchers cross-checked the results of the selected literature. If disagreements arose, they needed to be discussed with a third party. The Cochrane Evaluation Manual 5.3.3 was used as a benchmark to evaluate the quality of the subjects, including (1) random serial production; (2) distributed concealment; (3) blind method (patients, medical staff, outcome evaluation, and data analysis); (4) data integrity (tracking rate and important indicators); (5) selective reporting (hidden); (6) other sources of bias (such as baseline imbalance and suspected fraud). According to the above indicators, the two researchers' answer of “yes” indicated a lower risk of bias, “no” indicated a higher risk of bias, and “unclear” indicated an uncertain risk of bias.

### 2.4. Quantitative Data Synthesis

Meta-analysis was carried out using RevMan 5.3.3 software provided by Cochrane Collaboration Network. Relative risk (RR) and its 95% CI were used as combined effect quantities for counting data. Mean difference (MD) and its 95% CI were used as combined effect quantities for measuring data. Heterogeneity among the results was tested by*I*^2^test. When there was statistical homogeneity between the results (*P* > 0.1, *I*^2^ < 50%), the fixed effect model was used for meta-analysis; if there was statistical heterogeneity between the results (*P* < 0.1, *I*^2^ > 50%), the sources of heterogeneity were analyzed. If there was statistical heterogeneity between the two groups, there was no clinical heterogeneity or difference. The stochastic effect model was used for meta-analysis. If the heterogeneity between the results was too large, descriptive analysis was performed. Funnel charts were used to evaluate publication bias for outcomes involving more than 10 studies.

## 3. Results

### 3.1. Trial Flow and Study Characteristics

969 relevant literatures were initially detected from the relevant databases. According to the inclusion and exclusion criterion, 26 RCTs were included with 4676 patients in total consisting of 2342 cases of the experimental group and 2334 cases of the control group. Literature screening process and results were shown in Figure 1. Eighteen of the 26 studies included in the study were treated with JSBC plus other drugs, and eight trials were treated with JSBC plus basic drugs. Twenty-six studies were RCTs, which were included in the baseline characteristics table of the study as shown in Table 2.

### 3.2. Risk of Bias

Of the 26 studies included, all were judged as RCTs, of which 2 trials were randomly assigned according to random number table method; another two trials were randomly assigned according to the order of visits. All of them did not mention blind method and allocation concealment (Figure 2).

### 3.3. Meta-Analysis Outcome

#### 3.3.1. Urine Microprotein Excretion Rate UAER (ug/min)

Eighteen studies [6–9, 11, 13–17, 19, 23, 25, 27–31] analyzed the urinary microprotein excretion rate. The meta-analysis results showed that MD = −32.88, 95% CI (-48.35, -17.40), *P* < 0.0001, and *I*^2^ = 98%. This indicated that JSBC had significant difference in the treatment of diabetic nephropathy patients' urinary microprotein excretion rate (Figure 3).

#### 3.3.2. Serum Creatinine Scr Level

Sixteen studies [6–12, 14, 15, 20, 21, 23–27] were analyzed for serum creatinine. Meta-analysis showed that MD = −7.68, 95% CI (-10.96, -4.40), *P* < 0.0001, and *I*^2^ = 80%. There was a significant difference in the treatment of serum creatinine in diabetic nephropathy patients with JSBC (Figure 4).

#### 3.3.3. BUN Level

Thirteen studies [8–12, 14, 15, 20, 21, 24, 26–28] analyzed blood urea nitrogen (BUN). Meta-analysis showed that MD = −0.47, 95% CI (-0.72, -0.22), *P* = 0.0002, and *I*^2^ = 72%. It suggested that JSBC had significant difference in the treatment of BUN in patients with diabetic nephropathy (Figure 5).

#### 3.3.4. Urinary Albumin Level

11 studies [6, 7, 10, 12, 16, 20–22, 24, 26, 31] analyzed urinary albumin. Meta-analysis results showed that MD = −52.68, 95% CI (-77.78, -27.59), *P* < 0.0001, and *I*^2^ = 97%. It implied that JSBC had significant difference in the treatment of urinary albumin diabetic nephropathy patients (Figure 6).

#### 3.3.5. HbA1c (%) Glycosylated Hemoglobin

Seven studies [6, 8, 13, 16, 28, 29, 31] analyzed glycosylated hemoglobin. Meta-analysis showed that there was no significant difference in the treatment of glycosylated hemoglobin in patients with diabetic nephropathy by JSBC MD = −0.14, 95% CI (-0.03, -0.24), *P* = 0.02, and *I*^2^ = 3 (Figure 7).

#### 3.3.6. Fasting Blood Glucose FBG Level

Five studies [8, 11, 16, 29, 31] analyzed fasting blood glucose. Meta-analysis showed that MD = 0.18, 95% CI (-0.06, 0.42), *P* = 0.15, and *I*^2^ = 40%. There was no significant difference in the treatment of fasting blood glucose in diabetic nephropathy patients with JSBC (Figure 8).

## 4. Discussion

At present, there are few studies on JSBC in the treatment of diabetic nephropathy in China. In this paper, 26 studies were included to observe the core indicators of urinary microprotein excretion rate, urinary protein, glycosylated hemoglobin, BUN, serum creatinine, glycosylated blood sugar, and fasting blood sugar in patients with diabetic nephropathy. The current results suggested that protein excretion rate, urinary protein, glycosylated hemoglobin, blood urea nitrogen, serum creatinine, and other indicators have been improved, but the improvement of glycosylated hemoglobin and fasting blood sugar was not obvious.

Clinical medical trials have shown that diabetic patients are more likely to cause glomerulosclerosis on the basis of metabolic abnormalities and eventually lead to renal dysfunction [32–34]. High levels of chronic hyper glycaemia in diabetic patients lead to tissue hypoxia. The release of endothelin and nitrous oxide from endothelial cells can increase glomerular capillary tone, further leading to glomerular microangiopathy and thickening of the glomerular basement membrane. As the disease progresses, glomerulosclerosis eventually occurs and leads to renal failure [35–37].

JSBC is made by fermenting Cordyceps sinensis powder Cs-4. Cordyceps sinensis mycelium is considered as the most important component. Drug experiments have proved that Cordyceps sinensis mycelium contains a variety of amino acid trace elements, which has certain anti-inflammatory, kidney protection effects, and the lung-benefiting effect [38–40]. In recent years, a few of studies have shown that cystatin C (CysC) is an ideal serum marker reflecting glomerular filtration rate (GFR) with high sensitivity and specificity. It has been used in the diagnosis of early diabetic nephropathy [38]. It has been reported that Cordyceps preparation has a good therapeutic effect on diabetic nephropathy. Cordyceps preparation can correct the disorder of human fibrinolytic system and has a favorable therapeutic effect on early intervention of diabetic nephropathy. Cordyceps sinensis mycelium can reduce blood lipid faster. It can promote the rapid synthesis of liver and muscle proteins, improve the immune function of red blood cells, increase the blood supply of heart and brain, and inhibit platelet aggregation, which have a better protective effect on the functions of cardiovascular, cerebrovascular, hepatic, and renal systems [41].

It is worth mentioning that there are several important limitations in our meta-analysis. First, all RCTs were associated with high bias risk. To improve the quality of the trial, JSBC-related RCTs should be reported after the combination treatments of diabetic nephropathy in the future. Second, the test of system review was limited in China, and it needs to be further verified the application of other countries and regions. Third, all the studies included mentioned “randomness” without the mention blind methods or allocation concealment. There was a high risk of selective bias and measurement bias. Finally, the sample size in this study was small. The calculation of sample size should be considered when selecting randomized controlled trials in the future. There is therefore a need for larger, better designed, multicenter, randomized, double-blind trials in other countries.

## 5. Conclusions

The available clinical evidence has suggested that JSBC combined with western drugs is differentially effective in the treatment of diabetic nephropathy. The combination of JSBC with western medicine is more effective. However, due to the small amount and low quality of the included literatures, the current evidence is not certain to be fully clinically applicable. The efficacy benefits of the combination treatment are worthy of further study in the future.

## Figures and Tables

**Figure 1:** Literature screening process.

**Figure 2:** Risk of bias assessment of included studies. All of the 26 studies included did not mention blind method and allocation concealment.

**Figure 3:** Forest plot of urine microprotein excretion rate. This indicated that JSBC had significant difference in the treatment of diabetic nephropathy patients' urinary microprotein excretion rate.

**Figure 4:** Forest plot of serum creatinine Scr level. There was significant difference in the treatment of serum creatinine in diabetic nephropathy patients with JSBC.

**Figure 5:** Forest plot of BUN level. It suggested that JSBC had significant difference in the treatment of BUN in patients with diabetic nephropathy.

**Figure 6:** Forest plot of urinary albumin level. It implied that JSBC had significant difference in the treatment of urinary albumin diabetic nephropathy patients.

**Figure 7:** Forest plot of HbA1c glycosylated hemoglobin. There was no significant difference in the treatment of glycosylated hemoglobin in patients with diabetic nephropathy by JSBC.

**Figure 8:** Forest plot of fasting blood glucose level. There was no significant difference in the treatment of fasting blood glucose in diabetic nephropathy patients with JSBC.

**Table 1:** Search strategy in English and Chinese databases.

Search strategy in English and Chinese databases
1. Diabetes mellitus (mh)
2. Diabetes (mh)
3. Nephropathy (mh)
4. Diabetic nephropathy (mh)
5. Drinking and urine
6. Lower wasting-thirst
7. 1 or 2 or 3 or 4 or 5 or 6
8. Jinshuibao
9. Jinshuibao capsule
10. 8 or 9
11. Randomized controlled trial (pt)
12. Controlled clinical trial (pt)
13. Randomized (tiab)
14. Placebo (tiab)
15. Drug therapy (sh)
16. Randomly (tiab)
17. Trial (tiab)
18. Groups (tiab)
18. 11 or 12 or 13 or 14 or 15 or 16 or 16 or 17 or 18
19. Humans (mh)
20. 7 and 10 and 19
21. Animals (mh)
22. 21 not 22

**Table 2:** Summary of the randomized controls trials of JSBC for DN.

Study (author/year)	Sample size	Duration of treatment	Intervention group (regimen)	Control group (regimen)	Main outcomes	Intergroup differences
Higgins (2007) [5]	60 (30/30)	26 weeks	(A) JSBC, plus (B)	(B) Valsartan	24 h/UAlb; 8hUAER; HbA1c; ACR	24 h/UAlb: MD-, 140 [-227.65, -52.35] 8hUAER: MD, -32.17 [-48.68, -15.66] HbA1c: MD, -0.04 [-0.23.0.15] ACR: MD, -23.60 [-42.42, -4.78]
Dai (2016) [6]	90 (45/45)	30 weeks	(A) JSBC, plus (B)	(B) LPT, plus CT	24 h/UAlb; UAER; Scr; HbA1c	24 h/UAlb: MD, -36.6 [-44.14, -29.06] UAER: MD, -25.00 [-225.45, -200.55] Scr: MD, 0.90 [-3.04, 4.84] HbA1c: MD, 0.30 [0.08, 0.52]
Chen (2013) [7]	40 (20/20)	8 weeks	(A) JSBC, plus (B)	(B) LPT, plus CT	UAER; Scr; BUN; HbA1c	UAER: MD, -12.98 [-35.38 9.42] Scr: MD, -11.60 [-28.00, 4.80] BUN: MD, -1.40 [-2.11, -0.69] HbA1c: MD, 0.00 [-0.37, 0.37]
Yang (2014) [8]	40 (20/20)	12 weeks	(A) JSBC, plus (B)	(B) LPT, plus CT	UAER; Scr; BUN	UAER: MD, -25.19 [-31.24,-19.14] Scr: MD, -13.40 [16.93, -9.87] BUN: MD, -46.10 [-51.31, -40.89]
Zhang (2014) [9]	82 (49/33)	8 weeks	(A) JSBC, plus (B)	(B) Irbesartan, plus CT	Scr; BUN; 24 h/UAlb	Scr: MD, -16.6 [-22.72, -10.48] BUN: MD, -0.40 [-0.80, 0.00] 24 h/UAlb: MD, -47.20 [-72.82, -21.58]
Ding (2013a) [10]	100 (52/48)	2 weeks	(A) JSBC, plus (B)	(B) Irbesartan, plus CT	UAER; Scr; BUN	UAER: MD, -0.56 [-3.35, 53.73] Scr: MD, 8.03 [5.55, 10.51] BUN: MD, -0.46 [-1.90, 0.98]
Li and Yao (2009) [11]	70 (35/35)	12 weeks	(A) JSBC, plus (B)	(B) Irbesartan, plus CT	Scr; BUN; 24 h/UAlb	Scr: MD, -15.00 [-20.91, -9.09] BUN: MD, -1.40 [-2.11, 0.69] 24 h/UAlb: MD, -10.00 [-301.90, 281.90]
Yi et al. (2015) [12]	40 (20/20)	26 weeks	(A) JSBC, plus (B)	(B) Irbesartan, plus CT	UAER; HbA1c; ACR	UAER: MD, -24.20 [-40.32,-8.08] HbA1c: MD, -0.51 [-1.55,0.53] ACR: MD, -17.60 [=34.84, -0.36]
Shen et al. (2016a) [13]	60 (30/30)	8 weeks	(A) JSBC, plus (B)	(B) Candesartan cilexetil	UAER; Scr; BUN	UAER: MD, -17.93 [-27.56, -8.30] Scr: MD, -8.81 [-17.22, -0.40] BUN: MD, -0.17 [-1.04, 0.70]
Wu and Pan (2014a) [14]	68 (34/34)	8 weeks	(A) JSBC, plus (B)	(B) Candesartan cilexetil	UAER; Scr; BUN	UAER: MD, -19.66 [-29.90, -9.42] Scr: MD, -6.00 [-22.90, 10.90] BUN: MD, -0.10 [-1.54, 1.34]
Zhang et al. (2010) [15]	120 (64/56)	12 weeks	(A) JSBC, plus (B)	(B) Candesartan cilexetil, plus CT	UAER; 24 h/UAlb; HbA1c	UAER: MD, -14.60 [-38.17, 8.97] 24 h/UAlb: MD, -140.00 [-277.28,-2.72] HbA1c: MD, 0.13 [-0.05, 0.31]
Huang et al. (2010) [16]	64 (32/32)	8 weeks	(A) JSBC, plus PCI	(B) Perindopril, plus CT	UAER	UAER: MD, -28.47 [-34.17, -22.77]
Shi (2007) [17]	72 (37/35)	6 weeks	(A) JSBC, plus (B)	(B) Fosinopril, plus CT	UAER	UAER: MS, -29.80 [-35.68, -23.92]
Wang (2013) [18]	120 (60/60)	6 weeks	(A) JSBC, plus (B)	(B) Fosinopril, plus CT	UAER	UAER: MD, -28.13 [-32.57, -23.69]
Xiao et al. (2016) [19]	80 (40/40)	2 weeks	(A) JSBC, plus (B)	(B) Telmisartan, plus CT	Scr; BUN; 24 h/UAlb; ACR	Scr: MD, 1.60 [-2.84, 6.04] BUN: MD, -0.10 [-0.53, 0.33] 24 h/UAlb: MD, -40.30 [-50.63, -29.97] ACR: MD, -34.30 [-42.94, -25.66]
Pan and Shang (2010) [20]	60 (38/22)	13 weeks	(A) JSBC, plus (B)	(B) Benazepril, plus CT	Scr; BUN; 24 h/UAlb; ACR	Scr: MD, -1.80 [-8.67, 5.07] BUN: MD, 0.00 [-0.85, 0.85] 24 h/UAlb: MD, -100.00 [-119.84, -80.16] ACR: MD, -8.05 [-10.98, -5.12]
Wei (2013) [21]	80 (52/28)	8 weeks	(A) JSBC, plus (B)	(B) Olmesartan medoxomil, plus CT	24 h/UAlb; ACR	24 h/UAlb: MD, -100.00 [-119.84,-80.16] ACR:
Yu et al. (2017) [22]	106 (32/21)	12 weeks	(A) JSBC, plus (B)	(B) Atorvastatin, valsartan, plus CT	UAER; Scr	UAER: MD, -14.25 [-18.01, -10.49] Scr: MD, -14.25 [-18.01, -10.49]
Zhu and Li (2012) [23]	100 (50/50)	8 weeks	(A) JSBC, plus (B)	(B) CT	Scr; BUN; 24 h/UAlb	Scr: MD, 43.70 [-76.42, -10.98] BUN: MD, -1.50 [-2.07, -0.93] 24 h/UAlb: MD, -71.90 [-82.51, -61.29]
Gao (2010) [24]	50 (25/25)	26 weeks	(A) JSBC, plus (B)	(B) CT	UAER; Scr	UAER: MD, 5.36 [-23.26, 33.98] Scr: MD, 5.36 [-23.26, 33.98]
Jia et al. (2013b) [25]	60(30/30)	13 weeks	(A) JSBC, plus (B)	(B) CT	UAER; Scr; BUN	UAER: MD, -3.10 [-9.44, 3.24] Scr: MD, -3.10 [-9.44, 3.24] BUN: MD, -0.30 [-1.20, 0.42]
Li (2016b) [26]	120 (64/56)	4 weeks	(A) JSBC, plus (B)	(B) CT	Scr; BUN	Scr: MD, -4.34 [-8.27, -0.41] BUN: MD, -0.17 [-1.04, 0.70]
Wu et al. (2014b) [27]	60 (30/30)	12 weeks	(A) JSBC, plus (B)	(B) CT	UAER; Scr; BUN	UAER: MD, -1.60 [-16.03, 12.83] Scr: MD, -1.60 [-16.03, 12.83] BUN: MD, 0.10 [-1.36, 1.56]
Zhong and Guo (2006) [28]	60 (30/30)	8 weeks	(A) JSBC, plus (B)	(B) CT	UAER; HbA1c	UAER: MD, -18.70 [-27.58, -9.82] HbA1c: MD, -0.20 [-0.68, 0.28]
Liu (2009) [29]	60 (30/30)	12 weeks	(A) JSBC, plus CT	(B) Yishen Jiangtang mixture, plus CT	UAER; HbA1c	UAER: MD, 21.06 [11.53, 30.59] HbA1c: MD, 0.15 [-0.08, 0.38]
Wang et al. (2006) [30]	68 (34/34)	8 weeks	(A) JSBC, plus CT	(B) Lotensin, plus CT	UAER	UAER: MD, 0.74 [-9.18, 10.66]
Wang (2012) [31]	54 (27/27)	24 weeks	(A) JSBC, plus CT	(B) Shenling Baizhu powder, plus CT	24 h/UAlb; HbA1c	24 h/UAlb: MD, 39.49 [-3.40.82.38] HbA1c: MD, 0.07 [-0.37, 0.51]

## Data Availability

The datasets used and/or analyzed during the current study are available from the corresponding author on reasonable request.

## Abbreviations

JSBC: Jinshuibao capsule
DN: Diabetic nephropathy.
